# Application of Image Recognition Based on Wireless Sensors in Dance Teaching System

This article has been retracted.

**DOI:** 10.1155/2022/2440263

**Published:** 2022-06-01

**Authors:** Chi Ben

**Affiliations:** College of Wushu and Dance, Shenyang Sport University, Liaoning, Shenyang 110102, China

## Abstract

With the vigorous development of higher education in China, many universities have made great progress in various indicators in recent years. As the number of college students increases year by year, the effect of instruction in the classroom is especially important. The high quality of teaching directly affects the efficiency of students' listening to lectures, and more and more universities are receiving attention. However, the traditional dance classroom education and the one-to-many education model cannot adapt to the development trend of higher art education under the changes of the times and cannot effectively guarantee the quality of classroom education. The development of wireless sensor networks provides practical and feasible technical solutions for the development of dance education systems. Compared with general detection methods, image sensors can provide more real-time and more intuitive on-site information and wirelessly send image information to user terminals. This article describes the classic feature extraction algorithm and proposes a new feature extraction algorithm based on chart filling. The effectiveness of each algorithm is verified through several data sets. Image recognition is carried out by computer, including from computer to image processing, through the computer to recognize objects and various different modes of the target technology. The identification process usually includes several steps. First, the preprocessing of the image is required, then the segmentation of the image is performed, and then the feature extraction and matching are performed. In layman's terms, image recognition hopes to imitate the human heart to read photos. By applying the image recognition technology to the dance education system, changes in the methods and forms of dance education can be stimulated.

## 1. Introduction 

With the acceleration of the development of modern industrial society, the entire society has ushered in the trend of artificial intelligence [1]. People in all fields are beginning to take advantage of this opportunity to completely update the industry's old and backward technical methods. In the future, the power of the pioneers of reform will be brought into play. The same principle also applies to the field of distance network education [2]. In order to solve the problems in this field, the use of advanced artificial intelligence technology has become the consensus of scholars and experts in the 21st century [3]. First of all, the vast amount of information available on the Internet is the same as the way most students surf the Internet. The corresponding websites are browsed to obtain educational resources, and relevant databases are accessed to obtain teaching materials, etc. All these provide great motivation and opportunities for the development of distance education [4]. At present, Chinese school dance education still uses traditional learning methods. Education and education methods are still in the early stages of development, without information and digitization. In today's society, the development and education of school dance has the following modes: the first concept is to teach body language through language and behavior [5]. The previous education model was limited to face-to-face instruction, but this method allows the teacher to see the student's dance posture and details [6]. As time goes by, the student will immediately remember the details of the teaching and the teacher. Because each student's dance performance is not played repeatedly, its applicability is greatly restricted. The second is to download online. In this mode, students can download ready-made dance video resources directly from the Internet [7]. However, some websites have slower video updates and prolonged knowledge time. Students' learning progress will be slow, learning efficiency will be low, and college students' enthusiasm for learning will also be weakened. The third is to buy disks of teaching records. This model is similar to the purchase of dance video resources recorded by students. However, some disk resources are too old and will not be updated in a short time, so knowledge will have a long-time delay and the student's learning process will be interrupted, which is not helpful to learning.

At present, the establishment of a distance education network based on artificial intelligence technology and the use of embedded image recognition technology based on wireless sensor technology to form an efficient educational communication mode will help students form a better learning and communication atmosphere [8]. For teachers, it is also very simple to form a more concise teaching method and educational philosophy. However, in the teacher's curriculum, it takes a lot of time to prepare for related video recordings, dance education software learning, design concepts, and new technology updates. And, to solve the problem based on this, this article will design a set of remote online dance system to realize a multifunctional teaching system based on the B/S network structure [9]. The system has established a complete online learning and online interactive model database, which has improved the diversity of college dance teaching methods and teaching methods [10]. Moreover, the man-machine interface of the system is very convenient to use, and the login number of the teacher (in the case of the teacher), the login number of the student (in the case of the student), or the authentication login mode of unified ID is also adopted.

## 2. Related Work

According to the literature, the use of wireless sensors is mainly to perceive information about the environment or monitor objects in real time through microsensors [11]. Microsensors can not only work in simple equipment, low-cost, and harsh environments but also quickly capture the movements and movements of the monitored object [12]. The literature pointed out that after the distance education model taught by the Massachusetts Institute of Technology in the United States in the 1960s and 1970s was actively popularized in several European countries such as the United Kingdom and France, the promotion of practical applications, its practical application in the United States, and the nature of university education have a great influence all over the world. According to the literature, image recognition has been extensively studied and many recognition algorithms have emerged [13]. Feature extraction plays an important role in image recognition. In other words, the features that best represent the original data are extracted from the original data [14]. According to the literature, the graph embedding framework not only includes dimensionality reduction methods based on diversity learning but also includes dimensionality reduction algorithms that use linear methods such as locality and globalization [15]. These structures play a very important role in feature selection. According to the literature, China's online distance education started late and can be divided into three stages: communication education, radio and television education, and modern distance education [16].

## 3. Design and Implementation of the Embedded Image Recognition System Based on Wireless Sensors

### 3.1. System Principle and Architecture

The automatic sensor identification process is composed of operation unit, automatic identification rule reference, fault determination rule reference, and identification unit. The analog output signal of each sensor in the system is converted into a digital signal through the adjustment circuit and sent to the computer controller and calculation unit.

The operation unit extracts the feature quantity of the output signal of each sensor, and the extracted feature quantity includes arithmetic average, dispersion, range, difference, and variation period. The number of operation samples is 10–20. The number of samples that need to be drawn during the operation of the feature quantity is determined by the automatic identification rules. The automatic identification rule base and the fault judgment rule base are set before going offline according to the types and characteristics of the sensors used in the system. The rules contained on the basis of the two rules are based on professional knowledge, common sense knowledge, experience knowledge, etc.

According to the rules of the automatic recognition rule reference and the failure determination rule reference, the recognition unit automatically recognizes the characteristic quantity of each sensor output by the operation unit. It shall be determined whether the output of the identification unit will lead to the type, purpose, location, and absolute failure of the detection points used in the system. The automatic identification and fault determination steps must be executed after 15 minutes of operation of the central air-conditioning system.

The dance teaching system based on a wireless sensor network is composed of three parts: image sensing, image processing, and remote monitoring. The overall structure of the system is shown in Figure 1.

In Figure 1, the wireless transmission unit uses low-power wireless image sensor nodes to achieve on-site image acquisition, wireless transmission, and data reception. The image processing part is based on the ARM processor platform and image recognition algorithms to realize image preprocessing, feature extraction, and recognition. The remote monitoring part realizes remote communication through GPRS and the Internet. The wireless sending part of the online system is composed of several sensor nodes including image sensors, microprocessors, and wireless communication modules. Each node is divided into different clusters according to the region, and each member of the cluster sends data to the cluster source. The nodes in the cluster source select the appropriate path through a specific routing mechanism and send data to other cluster sources on the path. After multiple cluster sources are transmitted, the data set is sent to the sink node and the transmission process of the wireless network ends. Because the pixel value of the image cannot reflect the meaningful features of each image and distinguishing other meaningful features represented by low-level features is not strong, the convolution of the deep learning neural network is used to automatically learn the features of the deep image. If the image illustrates the characteristic significance feature, only the distance between the feature vectors of the image needs to be calculated and the similarity between the images can be judged based on the distance. Therefore, the application of deep learning neural network is an important part of the image retrieval system and the foundation of the entire system. The basic architecture of the AlexNet model of the convolutional neural network model used in this article is 8 layers, of which 5 layers are convolutional layers and 3 layers are fully integrated layers. The CIFAR-10 data set is selected as the image data set for training.

In an image search system, if the extracted image features are compared with the feature vectors of many images in the database, an unacceptable time cost will be incurred. Using the joint inversion indexing method to create a complementary inversion list between image feature vectors can not only narrow the scope of the search image but also greatly improve the efficiency of online search.

A series of candidate lists are visualized by comparing the query image and the combined inverted features. After calculating the hash code, not only can the calculation speed of the feature vector similarity be improved, but also the system storage space can be saved to a certain extent.

### 3.2. Image Processing Algorithm

#### 3.2.1. Image Embedding Framework

Compared with selecting the value of *k*, it is more difficult to select the value of *ε*. Therefore, *k* nearest neighbors are mostly used when constructing the graph and then the Gaussian kernel or 0-1 method is used to calculate the weight between samples, which is defined as follows.

In the Gaussian kernel, *P* is the similarity matrix between samples.

(1) $$\begin{array}{c} P_{ij}=\left\{\begin{array}{cc} \frac{\exp\left(-\left\|x_{i}-x_{j}^{2}\right\|\right)}{2\sigma^{2}}, & x_{j}\text{ is }x_{i}k\text{ nearest neighbors,}\\ \text{0,} & \text{other.} \end{array}\right) \end{array}$$

In the 0-1 method, *P* is the similarity matrix between samples.

(2) $$\begin{array}{c} P_{ij}=\left\{\begin{array}{cc} 1, & x_{j}\text{ is }x_{i}k\text{ nearest neighbors,}\\ 0, & \text{other.} \end{array}\right) \end{array}$$

The objective function of PCA is defined as follows:

(3) $$\begin{array}{c} \underset{W^{T}W=I}{\max}\sum_{i=1}^{n}{\left\|y_{i}-\bar{y}\right\|}^{2}. \end{array}$$

By deriving formula (3), we can obtain the following equation:

(4) $$\begin{array}{c} \underset{W^{T}W=I}{\max}tr\left(W^{T}SW\right). \end{array}$$

The objective function of LDA is

(5) $$\begin{array}{c} \max\frac{\sum_{i=1}^{C}n_{i}{\left\|W^{T}\mu_{i}-W^{T}\mu \right\|}_{2}^{2}}{\sum_{i=1}^{C}\sum_{x_{j\in c_{i}}}{\left\|W^{T}x_{j}-W^{T}\mu_{i}\right\|}_{2}^{2}}. \end{array}$$

We organize this to get

(6) $$\begin{array}{c} \underset{W}{\max}\frac{tr\left(W^{T}S_{b}W\right)}{tr\left(W^{T}S_{w}W\right)}. \end{array}$$

The objective function of LLE is

(7) $$\begin{array}{c} \underset{y}{\min}\varepsilon \left(y\right)=\sum_{i=1}^{N}{\left\|y_{i}-\sum_{j=1}^{k}W_{ij}y_{i}\right\|}^{2}. \end{array}$$

The solution method is

(8) $$\begin{array}{c} \left\{\begin{array}{cc} \underset{w}{\min}\varepsilon \left(w\right) & ={\sum_{i=1}^{N}\left\|x_{i}-\sum_{j=1}^{k}W_{ij}x_{j}\right\|}^{2}\\ s.t. & \sum_{j=1}^{k}W_{ij}=1 \end{array}.\right) \end{array}$$

We have,

(9) $$\begin{array}{c} \underset{w}{\min}\varepsilon \left(w\right)=\sum_{i=1}^{N}W_{i}^{T}S_{i}W_{i}. \end{array}$$

We use the Lagrangian multiplier method to solve equation (9), namely,

(10) $$\begin{array}{c} \Phi \left(W,\lambda \right)=\sum_{i=1}^{N}W_{i}^{T}S_{i}W_{i}-\lambda \left(\sum_{j=1}^{k}W_{ij}-1\right). \end{array}$$

#### 3.2.2. Image Local Discriminant Projection Feature Extraction

The projection of the local discriminant embedding is defined as follows:

(11) $$\begin{array}{c} W_{ij}=\left\{\begin{array}{cc} \exp\left[\frac{-{\left\|x_{i}-x_{j}\right\|}^{2}}{t}\right], & 1_{i}=1_{j},x_{i}\in N_{w}\left(x_{j}\right)\text{ or }x_{j}\in N_{w}\left(x_{i}\right)\\ 0, & \text{otherwise,} \end{array}\right.\\ W_{ij}^{\prime }=\left\{\begin{array}{cc} \exp\left[\frac{-{\left\|x_{i}-x_{j}\right\|}^{2}}{t}\right], & 1_{i}\neq 1_{j},x_{i}\in N_{b}\left(x_{j}\right)\text{ or }x_{j}\in N_{b}\left(x_{i}\right)\\ 0, & \text{otherwise.} \end{array}\right. \end{array}$$

According to the chart embedding theory, it is expected that the close relationship between the samples will be maintained after projection.

(12) $$\begin{array}{c} S_{w}=\sum_{ij}{\left\|P^{T}x_{i}-P^{T}x_{j}\right\|}^{2}W_{ij}=2tr\left\{P^{T}X\left(D-W\right)X^{T}P\right\},\\ S_{b}=\sum_{ij}{\left\|P^{T}x_{i}-P^{T}x_{j}\right\|}^{2}W_{ij}^{\prime }=2tr\left\{P^{T}X\left(D{}^{\prime }-W{}^{\prime }\right)X^{T}P\right\}. \end{array}$$

The goal of LDEP is to find the projection matrix *P* that maximizes the interclass dispersion and minimizes the intraclass dispersion. This can be expressed as the following optimization problem:

(13) $$\begin{array}{c} \underset{p}{\max}\frac{S_{b}}{S_{w}}=\frac{tr\left\{P^{T}X\left(D{}^{\prime }-W{}^{\prime }\right)X^{T}P\right\}}{tr\left\{P^{T}X\left(D-W\right)X^{T}P\right\}}. \end{array}$$

In order to completely reflect the differences of samples of different categories during the reconstruction of samples, the following conflict coordination representation learning model can be established for each training sample *x*_*i*_:

(14) $$\begin{array}{c} \underset{w_{i}}{\min}\left\{{\left\|x_{i}-Xw_{i}\right\|}_{2}^{2}+\lambda {\left\|w_{i}\right\|}_{2}^{2}+\lambda_{1}\sum_{c=1}^{C}{\left\|x_{i}-X_{c}w_{i}^{c}\right\|}_{2}^{2}\right\}. \end{array}$$

The optimal solution of *w*_*i*_ is obtained by seeking the partial derivative of equation (14) as follows:

(15) $$\begin{array}{c} w_{i}^{*}=\left(1+\lambda_{1}\right){\left(X^{T}X+\lambda I+\lambda_{1}M\right)}^{-1}X^{T}x_{i}, \end{array}$$

where *M* is defined as follows:

(16) $$\begin{array}{c} M=\left[\begin{array}{ccc} X_{1}^{T}X_{1} & \cdots & 0\\ \vdots & \ddots & \vdots \\ 0 & \cdots & X_{C}^{T}X_{C} \end{array}\right]. \end{array}$$

This paper defines the similarity weight matrices *U* and *U*′ of compact graphs within a class and separation graphs between classes, and the two matrix elements are defined as follows:

(17) $$\begin{array}{c} U_{ij}=\left\{\begin{array}{cc} w_{ij}^{*}, & \text{if }1_{i}=1_{j},\text{ and }w_{ij}^{*}>0,\\ \text{0,} & \text{other,} \end{array}\right.\\ U_{ij}^{\prime }=\left\{\begin{array}{cc} w_{ij}^{*}, & \text{if }1_{i}=1_{j},\text{ and }w_{ij}^{*}>0,\\ \text{0,} & \text{other.} \end{array}\right. \end{array}$$

According to the weight matrix of the compact graph within the class and the separation graph between classes, the following interclass separation is defined:

(18) $$\begin{array}{c} \sum_{i=1}^{n}\sum_{j=1}^{n}{\left\|P^{T}x_{i}-P^{T}x_{j}\right\|}^{2}U_{ij}=tr\left(P^{T}{\bar{S}}_{w}P\right),\\ \sum_{i=1}^{n}\sum_{j=1}^{n}{\left\|P^{T}x_{i}-P^{T}x_{j}\right\|}^{2}U_{ij}^{\prime }=tr\left(P^{T}{\bar{S}}_{b}P\right). \end{array}$$

Among them, ${\bar{S}}_{w}$ and ${\bar{S}}_{b}$, respectively, represent the compactness matrix within the class and the separability matrix between the classes, namely,

(19) $$\begin{array}{c} {\bar{S}}_{w}=\sum_{i=1}^{n}\sum_{j=1}^{n}\left(x_{i}-x_{j}\right){\left(x_{i}-x_{j}\right)}^{T}U_{ij}=X\left(D-H\right)X^{T},\\ {\bar{S}}_{b}=\sum_{i=1}^{n}\sum_{j=1}^{n}\left(x_{i}-x_{j}\right){\left(x_{i}-x_{j}\right)}^{T}U_{ij}^{\prime }=X\left(D{}^{\prime }-H{}^{\prime }\right)X^{T}. \end{array}$$

The diagonal elements are

(20) $$\begin{array}{c} D_{ii}=\sum_{j=1}^{n}U_{ij}+\sum_{j=1}^{n}U_{ji},\\ D_{ii}^{\prime }=\sum_{j=1}^{n}U_{ij}^{\prime }+\sum_{j=1}^{n}U_{ij}^{\prime }. \end{array}$$

The purpose of the local discriminant projection method based on the competitive coordination representation is to find the best projection matrix. In this way, the separation between the projected sample classes becomes larger, and the compactness within the classes becomes the smallest. In other words, the optimization model is as follows:

(21) $$\begin{array}{c} \underset{P}{\max}\frac{tr\left(P^{T}{\bar{S}}_{b}P\right)}{tr\left(P^{T}{\bar{S}}_{w}P\right)}. \end{array}$$

We solve $\;{\bar{S}}_{b}P=\lambda {\bar{S}}_{w}P$.

### 3.3. Simulation Results and Analysis of Image Recognition

#### 3.3.1. Analysis of Experimental Parameters

Starting from Table 1, if the values of *λ* and *λ*1 in the FERET data set are different, the recognition rate of CCRLDP will hardly fluctuate and will be relatively stable.

As shown in Table 2, when the recognition rate is the highest, the value of *λλ*_1_is very small, indicating that the competitiveness of the AR data set plays a small role.

It can be seen from Table 3 that as the value of *λ*1 increases, the overall recognition rate will increase accordingly. This is in the process of feature extraction, taking into account the competitiveness of all types of samples and the ability to judge. However, if the value increases to a certain value, the recognition rate will begin to decrease.

#### 3.3.2. Experimental Results

CCRC is a classification algorithm. The coefficients can be obtained directly through test samples. However, if the size of the input image is large, the complexity of the algorithm is particularly high.  Table 4 shows the algorithms for calculating time with various data sets in most cases. In some cases, the calculation speed of this paper is faster than other algorithms and the calculation time of the specific algorithm is less, but the recognition rate is much lower than the algorithm of this paper.

Figures 2–4 show the average recognition rate of five different algorithms other than the CCRC algorithm, and the recognition rate on the noisy FERET is shown in Figure 2. The curves vary according to the dimension of the feature space of each data set (CCRC directly classifies the original data of the test set because it does not involving feature extraction; that is, there is no size change problem).

The recognition rate on Binalpha is shown in Figure 3.

The trend graph of the recognition rate of different algorithms on each data set as the number of features increases is shown in Figure 4.

## 4. Computer-Aided Dance Teaching System Application and Innovation Research

### 4.1. The Overall Design Scheme of System Function

Figure 5 shows the specific and complete function architecture diagram of the remote online burning system. This diagram is actually a more specific functional representation after merging the corresponding modules of teachers, students, and administrators. For example, the teacher's functions are divided into management software and video, management resource evaluation, management test, management homework, upload, and download. Students are divided into forum discussion, query results, course selection, video display, etc.

The design principles and purposes of the online dance teaching system mainly cover 8 aspects: economy, safety, scalability, height, reliability, practicability, simplicity, and hierarchical modularity. These are analyzed and explained in detail as follows: the two main architectures of software technology are C/S architecture and B/S architecture. The C/S (client/server) architecture is a client/server architecture, which is widely used in the current software technology architecture. There used to be two-tier and three-tier C/S architecture; the most classic is the two-tier C/S architecture. The B/S (browser/server) architecture is a browser/server architecture, which is a relatively new software system for constructing the architecture. The traditional C/S architecture cannot meet the existing Internet global network interconnection and open requirements. The globalization trend and the increasingly popular B/S structure have changed the traditional architecture system, providing software developers with new ways of thinking and having a more innovative structure. The specific functional architecture diagram of the remote online dance teaching system is shown in Figure 5.

### 4.2. Database Table Design

#### 4.2.1. Teacher Information Form

The teacher information table is mainly used to save the relevant information of the teacher, such as the teacher's name, age, salary number, password, teacher's gender, birthday, teacher's work unit, professional teacher, research institute, research direction, teacher title, teacher's location, postgraduate number, work of spouse, teacher's courses, and number of courses this semester. The specific teacher data table information is shown in Table 5.

#### 4.2.2. Student Information Form

The function of the student information table is to save the student's name, age, login password, gender, birthday, college student, expert student, submitted class, and other student related information, as well as the number of people who join the school community and school group, whether to join the club and its number, and the selection of elective subjects and courses. The specific student data table information is shown in Table 6.

#### 4.2.3. Video Upload Management Information Table

Video upload management information table is mainly used to upload video type, video start time, video end, dance video classification (belonging to classical dance, international standard dance, dance, ethnic, and ballet), and other related video information, videos, voice clips, number of all uploaded videos, video title, video producer, dance, and story format of dance theme. Specific video upload management information is shown in Table 7.

#### 4.2.4. Courseware Upload Management Table

The management information table for uploading courseware is mainly used for uploading relevant information of courseware software. Among them are the type of uploaded courseware, the time and classification of the uploaded courseware, the number of all uploaded courseware, the name of the courseware, the production of the courseware, the subject and the space occupied by the courseware software, the size (*M*), the chapters of the corresponding textbook, the audit of the failed courseware, the number of inspections that did not pass the courseware software, the number of inspections that did not pass the courseware software, and the number of inspections that passed the courseware software. The specific video upload management information is shown in Table 8.

#### 4.2.5. Submit Job Information Form

The homework submission information form is mainly for students submitting homework-related information. It mainly includes the following content, assignment number, number of assignments submitted, assignment questions, work completion timetable in writing, assignments submitted to the author, work submission time, file name, work number, assignments occupying pages corresponding to the size of the textbook space, and the performance level of homework exercises and homework. The specific job information submitted is shown in Table 9.

#### 4.2.6. Publish Job Information Table

The release task information table is mainly used for the release of teacher information. It mainly includes the following contents: public assignment number, number of assignments, post assignment processing questions, teacher response completion, assignments, assignment time, post statistical assignment file names, assignment answers, solving difficult assignment problems, and post corresponding tests. The specific release task information is shown in Table 10.

#### 4.2.7. Course Information Form

The course information table is mainly used to display the course information platform, such as course number, course name, number of selected courses, course summary content, number of course selections, course introduction, number of innovative courses, and course attributes. The specific course information is shown in Table 11.

### 4.3. Innovative Strategies for Computer-Assisted Dance Teaching Courses

The 3D assistant system of the dance creation computer is the concept of digital dance. This is a dance choreography software system based on the 3DS Max system and the main development platform, using physical simulation of objects moving in the field of 3D graphics and various material rendering techniques. Based on the powerful 3D software 3DS Max, the operation and labor-saving have the advantages of convenient, realistic, intuitive demonstration, quick response, and simple correction simulation. One must optimize and edit the dance moves of the existing dance movement database and finally confirm the finished product of 3D visual dance. This technology has a very high value, that is, to establish the prospects of the field and the extension of the field. As a new technology, the dance creation computer-aided three-dimensional system can meet the special requirements of making digital dances. Through its convenient use method, students can progress according to their creative intentions. In order to improve learning efficiency and speed, in order to design satisfactory works, relevant standards will be formulated and revised continuously to achieve the goal. Therefore, it is necessary to use big data thinking for teaching design. First, we must scientifically formulate teaching goals. The teaching design is based on the further development of the teaching goal. The dance teaching goal has not changed from a large level. However, with the development of the times, we have many different needs for many detailed contents. After refining the teaching goals, how to scientifically and accurately determine the teaching goals of each knowledge point is a key step to improve the quality of dance teaching. The teaching goals determined through personal subjective consciousness and experience and lessons are not supported by data and, to a certain extent, are unconvincing. We must analyze the complex big data information and use the results reflected by the data to formulate teaching goals based on the data, so that teaching is more scientific and accurate. Applying the principle of big data precision to the teaching of dance and by tracking the teaching trajectory of the teacher, the learning trajectory of the student, and the interactive data between the two, the teaching characteristics of the teacher, the learning characteristics of the students, and the psychological characteristics of the students are obtained. The characteristics of different objects are accurately presented, and then, teaching decisions are implemented to scientifically determine the teaching goals of dance, promote the formulation of teaching goals more scientifically, more in line with the needs of current student development, and better realize the precise teaching of dance lessons. The second point is to choose the teaching content scientifically. Big data technology is a product of the development trend of informatization, and its wide application promotes the transformation of college dance teaching thinking from perceptual qualitative analysis to rational quantitative analysis. In traditional dance teaching, teachers often teach courses based on long-term teaching experience. Now, the application of big data technology in dance classes has greatly improved this situation. Using big data to transform teaching thinking, one must change the qualitative analysis teaching thinking based on teachers' perceptual cognition and form a rational quantitative analysis teaching thinking based on student needs, which is conducive to enhancing the effectiveness of dance lessons.

As a system that can break the original choreography guidance model, the computer-assisted three-dimensional dance production system displays the effects of students' creative ideas in the form of rehearsal and guides choreography, which can provide a realistic and visible platform. Students use the three-dimensional computer-aided system to call the actor pictures designed in the database according to their own artistic concepts, create various role dance works required for choreography, imitate dance action data, and imitate dance performers. In this way, the synthesis and transformation of body language, the scheduling model of dance posture, the formation and composition of space, and the overall framework of change are carried out. At the same time, because of its multiple values, artistic creation can also strengthen students to learn the skills of choreographers.

Interest is the biggest motivation for learning through the computer's 3D assistance system. Through this method, students can continuously practice the skills of the choreographer independently, combine the charm of dance choreography, feel the essence of composition, and improve it. Students' desire to learn, participate in artistic creation, and develop creative thinking can ultimately improve and perfect their creative desire and creative concept in the process of choreography and performance.

The computer's 3D assistant system can effectively guide the choreography, and it is important to establish a database. In the dance movement, the use of motion capture technology can capture various dance movements of professional actors from all parts. From all angles of the body, a three-dimensional image is established to make it easier to use in education. Regarding character images, the height, age, clothes, skin, hair style, decorations, and other contents of various characters need to be stored in the database. These contents must be consistent with the style and content of the dance. In addition, in performance environments such as lighting, stage, curtains, and smoke, only the construction of a rich database can meet the needs of education.

The application of the computer 3D assistant system has played a positive role in guiding education. Teachers can accurately show the director's application of various skills through intuitive, clear, and vivid photos. Students may be personally influenced, so the imperceptible education will deepen thinking, understanding, and memory of educational content, but independent operations such as learning to use can improve the ability of guidance. As a tool and platform for optimizing projects, it shows that choreography teaching can develop faster and better. As a creative idea of education reform, the combination of dance and modern advanced technology reflects the current new level of education.

## 5. Conclusion

In recent years, science and technology have developed rapidly, and a large amount of data has emerged in various industries, including more and more image data. However, images generally have a high dimensionality, and the complexity of data processing is too high. Traditional data analysis and processing have been difficult to cope with. With the higher dimensional data, the role of data dimensionality reduction is becoming more and more important. The dimensionality reduction algorithm based on the graph embedding framework plays an important role. The research object of this article is the application of the image embedding theory in the dance teaching system and the innovation strategy of dance teaching courses. With the help of the latest information technology, the traditional classroom teaching mode can be converted into the Internet and a new online dance instruction mode can be realized. Based on the existing education system, platform, and the corresponding latest programming methods and database technology, this thesis realizes the flexible education of dance courses and thus proposes an online distance education system that popularizes the concept and mechanism of distance education.

## Figures and Tables

**Figure 1:** The overall structure of the system.

**Figure 2:** The recognition rate on the noisy FERET.

**Figure 3:** Recognition rate on Binalpha.

**Figure 4:** The trend of the recognition rate of different algorithms on each data set as the number of features increases: (a) the recognition rate of 10 × 10 occlusion AR and (b) the recognition rate of 15 × 15 occlusion AR.

**Figure 5:** The specific functional architecture diagram of the remote online dance teaching system.

**Table 1:** Comparison of FERET data set parameters.

*λλ*_1_	0.001	0.01	0.1	1	10	100
0.001	73.41	70.34	71.23	73.66	76.05	73.65
0.01	73.06	70.59	72.02	74.09	74.85	73.59
0.1	72.59	71.26	71.56	75.28	74.59	74.76
1	71.52	71.23	73.69	75.31	74.05	75.65
10	75.16	69.01	74.59	76.51	74.90	75.09
100	74.93	73.40	73.48	75.48	73.31	74.55

**Table 2:** Comparison of AR data set parameters.

*λλ*_1_	0.001	0.01	0.1	1	10	100	1000
0.001	90.71	90.72	87.91	83.31	83.85	81.79	84.45
0.01	90.45	89.59	88.38	84.75	84.54	83.95	83.32
0.1	89.65	89.75	88.21	84.28	81.70	83.74	82.95
1	91.21	89.76	87.74	85.68	82.79	83.43	84.38
10	90.63	90.66	87.77	84.52	82.24	84.31	81.71
100	90.52	90.94	88.37	85.68	82.99	82.86	82.27

**Table 3:** Comparison of Binalpha data set parameters.

*λλ*_1_	0.001	0.01	0.1	1	10	100	1000
0.001	64.72	70.72	72.22	79.28	82.41	83.65	81.70
0.01	66.15	69.75	73.23	80.01	83.28	82.52	81.34
0.1	65.87	70.33	74.34	77.87	82.05	72.14	81.41
1	82.75	70.75	73.68	79.05	82.23	82.11	81.78
10	72.55	74.19	76.89	79.91	80.15	81.92	83.25
100	78.37	76.39	78.37	81.62	82.53	82.45	81.72
1000	79.70	80.53	81.25	84.25	82.54	83.40	81.53

**Table 4:** Calculation time (s) of each algorithm on different data sets.

Data set	LPP	CRP	CRRP	CCRC	CRLDP
FERET (*L* = 5)	1.6392	2.3495	2.5917	1.0464	1.7126
AR (*L* = 12)	3.1276	31.1444	42.072	10.1262	27.0833
Binalpha (*L* = 20)	2.1103	73.9823	10.8593	4.3503	1.8114

**Table 5:** Teacher information table.

Field definition	Field type	Field description
Teacher_ID	Long	Object identifier
Teacher_Name	Varchar	Teacher's name
Teacher_Age	Int	Teacher's age
Teacher_Number	Int	Pay slip number
Teacher_Password	Varchar	Login password
Teacher_Sex	Varchar	Teacher gender
Teacher_Birthday	Datetime	Teacher's birthday
Teacher_Academy	Varchar	Teacher's college
Teacher_Profession	Varchar	Teacher's major
Teacher_Institute	Text	Teacher's institute
Teacher_ResearchFocus	Text	Research direction
Teacher_TechnicalPost	Varchar	Teacher title
Teacher_Position	Varchar	Teacher position
Teacher_SpouseJob	Varchar	Spouse work
Teacher_Course	Varchar	Teacher's course
Teacher_CourseNumbers	Int	Number of courses taught by teachers in this semester

**Table 6:** Student information sheet.

Field definition	Field type	Field description
Student_ID	Long	Object identifier
Student_Name	Varchar	Student name
Student_Age	Int	Student age
Student_Number	Double	Student ID
Student_Password	Varchar	Login password
Student_Sex	Varchar	Student gender
Student_Birthday	Datetime	Student birthday
Student_Academy	Varchar	Student's college
Student_Profession	Varchar	Student's major
Student_ClassPosition	Varchar	Class position
Student_SchoolOrgan	Varchar	Join the school's club
Student_SchoolOrganNum	Int	Number of school clubs joined
Student_OptionalCourse	Varchar	Elective course selection
Student_OptionalCourseN	Int	Number of elective courses selected

**Table 7:** Video upload management information table.

Field definition	Field type	Field description
Video_ID	Long	Object identifier
Video_Type	Varchar	Uploaded video type
Video_Starttime	Datetime	Video start time
Video_Endtime	Datetime	Video end time
Video_Audio	Varchar	Video sound clip
Video_Allnumbers	Int	Number of all uploaded videos
Video_Name	Varchar	Video name
Video_Producer	Varchar	Video producer
Video_Dancename	Varchar	Dance name
Video_Story	Text	Dance story
Video_Topic	Text	Dance theme
Video_Form	Varchar	Dance performance

**Table 8:** Courseware upload management information table.

Field definition	Field type	Field description
Courseware_ID	Long	Object identifier
Courseware_Type	Varchar	Upload courseware type
Courseware_Time	Datetime	Courseware upload time
Courseware_classification	Int	Courseware classification
Courseware_Numbers	Int	Number of all uploaded courseware
Courseware_Name	Varchar	Courseware name
Courseware_Producer	Varchar	Courseware producer
Courseware_Topic	Text	Courseware theme
Courseware_Space	Int	The space occupied by the courseware (M)
Courseware_Section	Varchar	Textbook chapters corresponding to the courseware
Courseware_Nopass	Int	Number of failed courseware
Courseware_Pass	Int	Number of approved courseware
Courseware_Nopasscourse	Varchar	Review failed courseware
Courseware_Passcourse	Varchar	Approved courseware

**Table 9:** Submit job information form.

Field definition	Field type	Field description
Homework_ID	Long	Number of the submitted job
Homework_Numbers	Int	Number of submissions
Homework_Complete	Varchar	Homework completion progress
Homework_Author	Varchar	Assignment submission author
Homework_Time	Date time	Assignment submission time
Homework_Filename	Varchar	Job file name
Homework_Nums	Text	Assigned job number
Homework_Space	Int	The amount of space occupied by the job
Homework_Degrade	Int	Homework correction scoring grade
Homework_Selfrevised	Bool	Whether the assignment is corrected by yourself

**Table 10:** Post job information table.

Field definition	Field type	Field description
Homeworkissue_ID	Long	Number of the posted job
Homeworkissue_Numbers	Int	Number of job postings
Homeworkissue_Author	Varchar	Statistics of job response
Homeworkissue_Time	Datetime	Assignment correction time
Homeworkissue_Filename	Varchar	Job file name published
Homeworkissue_Answer	Text	Homework answer
Homeworkissue_Hard	Int	Difficulty of homework
Homeworkissue_Test	Int	The published assignments correspond to the exam questions

**Table 11:** Course information table.

Field definition	Field type	Field description
Class_ID	Long	Course no.
Class_Name	Varchar	Course title
Class_Numbers	Int	Number of courses available
Class_Content	Varchar	Course summary content
Class_Stunumbers	Int	Number of students choosing courses
Class_Brief	Text	Course introduction
Class_Innovate numbers	Int	Number of innovative courses
Class_Properties	Varchar	Course attributes

## Data Availability

No data were used to support this study.
